# Discrimination of urinary exosomes from microvesicles by lipidomics using thin layer liquid chromatography (TLC) coupled with MALDI-TOF mass spectrometry

**DOI:** 10.1038/s41598-019-50195-z

**Published:** 2019-09-25

**Authors:** Nilubon Singhto, Arada Vinaiphat, Visith Thongboonkerd

**Affiliations:** Medical Proteomics Unit, Office for Research and Development, Faculty of Medicine Siriraj Hospital, Mahidol University, Bangkok, 10700 Thailand

**Keywords:** Multivesicular bodies, Lipidomics, Isolation, separation and purification, Lipids, Kidney

## Abstract

Urinary extracellular vesicles (EVs), including microvesicles and exosomes, play several important roles in cell biology and serve as potential biomarkers in various kidney diseases. Although they have differential biophysical properties, specific biomarkers are required to discriminate these EVs during isolation/purification. The present study aimed to define differential lipidome profiles of urinary microvesicles vs. exosomes. Urine samples collected from eight healthy individuals were pooled and underwent lipid extraction using 2:1(v/v) chloroform/methanol. The recovered lipids were resolved by thin layer liquid chromatography (TLC) and analyzed by MALDI-TOF MS. From three and five TLC bands observed in microvesicles and exosomes, respectively, several fatty acids, glycerolipids and phospholipids were identified from both EVs without clear differential patterns. However, their sphingolipid profiles were unique. Ceramide phosphates (CerP), hexosyl sphingoid bases (HexSph), lactosyl ceramides (LacCer), mannosyl di-PI-ceramides (M(IP)2 C), sulfatides hexosyl ceramide (SHexCer) and sulfatides hexoxyl sphingoid bases (SHexSph) were detectable only in urinary exosomes, whereas phosphatidylinositol ceramides (PI-Cer) were detectable only in urinary microvesicles. The presence of CerP only in urinary exosomes was successfully validated by dot blot analysis. Our extensive lipidome analyses of urinary microvesicles vs. exosomes provide potential lipidome markers to discriminate exosomes from microvesicles and may lead to better understanding of EVs biogenesis.

## Introduction

Extracellular vesicles (EVs) are the lipid-enclosed particles that can be found mainly in human body fluids, particularly urine^1^. Urinary EVs can reflect physiologic and pathologic states of the urinary system, e.g., from podocytes to renal tubular cells of the nephron. Therefore, EVs serve as the excellent source for studying the renal physiology and pathophysiology of kidney diseases^2^. There are two major types of EVs, including exosomes and microvesicles, that play several important roles in cell biology and serve as potential biomarkers in various kidney diseases^3^. These two types of EVs have some differential biophysical and biochemical properties, e.g., size, shape, density, and biomolecular components^4^. Exosomes are the nano-scale vesicles ranging from 30–120 nm with spherical or cup-like morphology, whereas microvesicles are in irregular shape and larger with a wide range of size up to approximately 1,500 nm (>10 times greater than that of exosomes)^4,5^.

Base on their biophysical and biochemical properties, current isolation protocols of exosomes and microvesicles (e.g., differential ultracentrifugation and OptiPrep kit) are based mainly on their sizes, densities and flotation velocities^6–8^. Other isolation protocols include immuno-affinity and solvent-based precipitation^6–8^. Nevertheless, the purity for isolation/purification of these two types of EVs remains the critical issue for their analyses. In addition, it is necessary to define precise markers for each of these two EVs that can be used for discriminating them during isolation/purification and for better understanding of their biology and functions. The present study aimed to define differential lipidome profiles of urinary microvesicles vs. exosomes using thin layer liquid chromatography (TLC) followed by matrix-assisted laser desorption/ionization time-of-flight mass spectrometry (MALDI-TOF MS). The identified distinct lipid species that could potentially be useful for discriminating them was finally validated by conventional immunoassay.

## Results

The present study employed TLC followed by MALDI-TOF MS for lipidome profiling of urinary microvesicles and exosomes to define lipid marker(s) to discriminate these two types of EVs for determining the purity of their isolation/purification. All experimental procedures in this study are summarized as a schematic workflow shown in Fig. 1. After isolation/purification, urinary microvesicles and exosomes were subjected to examination by transmission electron microscopy (TEM). The results showed that both of these urinary EVs were present as the typical membrane-bounded, spherical-shape vesicles with sizes of approximately 100 nm for microvesicles and 30–50 nm for exosomes (Fig. 2). The lipids were then extracted from both types of these urinary EVs. From 300 ml of the pooled urine, 3.08 ± 1.02 mg lipids were obtained from microvesicles, whereas 0.80 ± 0.19 mg lipids were yielded from exosomes. An equal amount of lipids (10 µg/sample) derived from each sample was then resolved by TLC. The data showed that TLC band patterns obtained from urinary microvesicles and exosomes were consistent in all four independent experiments. While microvesicles had few TLC bands present only at the top of the TLC lane, exosomes had the greater number of TLC bands visualized along the entire TLC lane (Fig. 3). These results indicated the distinct lipidome profiles of urinary microvesicles vs. exosomes.

**Figure 1:** Schematic workflow of all experimental procedures in this study. Urine samples were collected and microvesicles and exosomes were isolated/purified by differential centrifugation technique. Each of these two types of EVs was then subjected to lipid extraction using 2:1(v/v) chloroform/methanol. The extracted lipids were then resolved by thin layer liquid chromatography (TLC) and identified by MALDI-TOF MS. Differential lipid species that might serve as the potential markers to discriminate these two types of EVs was finally validated by a conventional method such as dot blot analysis.

**Figure 2:** Transmission electron microscopy (TEM). After isolation/purification, urinary microvesicles (**A**) and exosomes (**B**) were negatively stained by uranyl acetate and their images were captured by TEM (original magnification = 50,000×).

**Figure 3:** Consistent and distinct TLC lipidome profiles of urinary microvesicles vs. exosomes. After isolation/purification, lipids were extracted from urinary microvesicles and exosomes and then resolved by TLC. The data showed consistent TLC band pattern of each type of these two EVs in all four independent experiments. Moreover, the TLC band pattern of lipids derived from urinary microvesicles obviously differed from those derived from urinary exosomes. The full-length images of these cropped TLC plates are provided in Supplementary Fig. S1. MV = microvesicles; Exo = exosomes.

To further characterize the lipids extracted and recovered from urinary microvesicles vs. exosomes using the same extraction protocol, the TLC-resolved lipids were subjected to lipid identification/characterization by MALDI-TOF MS. The data revealed that each TLC band had a distinct MS spectral profile and each profile contained the spectra varying from 400–1700 *m/z* (Fig. 4). Interestingly, the MS spectral pattern of lipids derived from TLC Band1 of microvesicles (MV1) looked similar to that of the lipids derived from TLC Band1 of exosomes (Exo1). However, other TLC bands of lipids derived from microvesicles and exosomes obviously differed (Fig. 4).

**Figure 4:** MS profiling and identification of lipid species derived from urinary microvesicles vs. exosomes. Three TLC bands of lipids derived from urinary microvesicles and five of those derived from urinary exosomes were subjected to MALDI-TOF MS analysis. The MS spectra of each TLC band acquired by positive ionization mode in the *m/z* range of 0–2,000 are shown. MV = microvesicles; Exo = exosomes.

After profiling, all the *m/z* values of these lipid ions were searched against LIPID MAPS Structure Database (LMSD) using the LIPID MAPS tool (www.lipidmaps.org/tools). A total of 40 lipid species were identified from TLC Band1-Band3 of microvesicles (MV1-MV3) and TLC Band1-Band5 of exosomes (Exo1-Exo5), including those under sphingolipid, fatty acid, glycerolipid and phospholipid classes (Table 1) (see also Supplementary Tables S1 and S2). Examples for the assignment of each of the MS spectra to a specific lipid species are illustrated in Fig. 5 (in which the identifications of PG(44:11) from the *m/z* of 869.531 in MV1 band and PI(37:6) from the *m/z* of 869.509 in Exo1 band are demonstrated). Additionally, their spectral intensities were analyzed and the quantitative data are summarized in Fig. 6. From these qualitative and quantitative data, except only for mono(acyl|alkyl)glycerols (MG) that was found only in MV1 but not in any of the exosomal TLC bands, several fatty acids, glycerolipids and phospholipids were identified from both microvesicles and exosomes without clear differential patterns. Interestingly, their sphingolipid profiles were quite unique. Ceramide phosphates (CerP), hexosyl sphingoid bases (HexSph), lactosyl ceramides (LacCer), mannosyl di-PI-ceramides (M(IP)2 C), sulfatides hexosyl ceramide (SHexCer) and sulfatides hexoxyl sphingoid bases (SHexSph) were detectable only in urinary exosomes, whereas phosphatidylinositol ceramides (PI-Cer) were detectable only in urinary microvesicles (Table 1 and Fig. 6). Therefore, these unique lipid species found only in exosomes or microvesicles may be used as the markers to discriminate these two types of EVs.

**Table 1:** Summary of lipid species identified from individual TLC bands of urinary microvesicles and exosomes using MALDI-TOF MS.

Lipid class	Lipid species	Urinary microvesicles			Urinary exosomes				
		Band1 (MV1)	Band2 (MV2)	Band3 (MV3)	Band1 (Exo1)	Band2 (Exo2)	Band3 (Exo3)	Band4 (Exo4)	Band5 (Exo5)
Sphingolipid	Ceramides (Cer)	+	+	+	+	+	+	+	+
	Ceramide phosphates (CerP) *	−	−	−	+	+	+	+	+
	Hexosyl ceramides (HexCer)	+	+	+	+	+	+	+	+
	Hexosyl sphingoid bases (HexSph) *	−	−	−	−	−	+	−	+
	Lactosyl ceramides (LacCer) *	−	−	−	−	+	−	−	−
	Lactosyl sphingoid bases (LacSph)	+	+	−	+	−	+	+	−
	Mannosyl-di-PI-ceramides (M(IP)2 C) *	−	−	−	−	+	−	−	−
	Mannosyl-PI-ceramides (MIPC)	+	−	−	+	+	−	+	+
	Sphingomyelins (LysoSM)	+	+	+	−	−	−	+	+
	PE-ceramides (PE-Cer)	+	+	+	+	+	−	+	+
	PI-ceramides (PI-Cer) #	+	−	+	−	−	−	−	−
	Sulfatides hexosyl ceramide (SHexCer) *	−	−	−	−	−	−	−	+
	Sulfatides hexosyl sphingoid bases (SHexSph) *	−	−	−	−	+	+	+	+
	Sphingomyelins (SM)	+	−	+	−	−	−	+	−
Fatty acid	Acyl carnitines (CAR)	+	+	+	+	+	−	+	+
	Acyl CoA’s (CoA)	+	−	+	+	+	+	+	+
	Cardiolipins (CL)	+	−	−	+	−	−	−	−
	Cholesteryl esters (CE)	+	+	+	−	−	−	+	+
	Fatty acids (FA)	+	+	+	+	+	+	+	+
	Wax esters (WE)	+	+	+	+	+	+	+	+
Glycerolipid	Di(acyl|alkyl)glycerols (DG)	+	+	+	+	+	+	+	+
	Mono(acyl|alkyl)glycerols (MG) #	+	−	−	−	−	−	−	−
	Monogalactosyldiacylgylcerols (DGDG)	+	+	+	+	+	+	+	+
	Monogalactosyldiacylgylcerols (MGDG)	+	+	+	+	−	+	+	+
	Sulfoquinovosyldiacylglycerols (SQDG)	+	+	+	+	+	+	+	+
	Tri(acyl|alkyl)glycerols (TG)	+	+	+	+	+	+	+	+
Phospholipid	Lysophosphatidic acids (LPA)	+	+	−	+	+	−	+	+
	Lysophosphatidylcholines (LPC)	+	+	+	+	+	+	+	+
	Lysophosphatidylethanolamines (LPE)	+	+	+	+	+	−	+	+
	Lysophosphatidylglycerols (LPG)	+	+	+	+	+	+	+	+
	Lysophosphatidylinositols (LPI)	−	+	+	+	+	+	+	+
	Lysophosphatidylinositol phosphates (LPIP)	+	+	+	+	+	+	+	+
	Lysophosphatidylserines (LPS)	+	+	+	−	+	+	−	−
	Phosphatidic acid (PA)	+	+	+	+	+	+	+	+
	Phosphatidylcholines (PC)	+	+	+	+	+	+	+	+
	Phosphatidylethanolamine (PE)	+	+	+	−	+	−	−	−
	Phosphatidylglycerols (PG)	+	+	+	+	+	+	+	+
	Phosphatidylinositols (PI)	+	+	+	+	+	+	+	+
	Phosphatidylinositol phosphates (PIP)	+	+	+	+	+	+	+	+
	Phosphatidylserines (PS)	+	+	+	+	+	+	+	+

Symbols used: +Found; −Not found; *Present only in exosomes; ^#^Present only in microvesicles.

**Figure 5:** Illustration of the assignment of each MS spectrum to a specific lipid species. The zoom-in images show the MS spectra in the *m/z* range of 850–900 and the spectra at the *m/z* 869.531 in MV1 and *m/z* 869.509 in Exo1 bands were identified as PG(44:11) and PI(37:6), respectively.

**Figure 6:** Quantitative analysis of mass spectral intensity of each identified lipid species. Each bar represents mean relative intensity of each lipid species normalized by total intensity of all lipids identified in each sample. * = the lipid species that were detectable only in urinary exosomes; # = the lipid species that were detectable only in urinary microvesicles; MV = microvesicles; Exo = exosomes.

From these differential unique lipid species, CerP drew our attention because it was consistently found in all TLC bands of urinary exosomes (Exo1-Exo5) (Table 1 and Fig. 6). Dot blot analysis was thus performed to validate this lipidomics finding. The dot blot data showed that CerP was consistently found in urinary exosomes but was not detectable in urinary microvesicles in all three independent experiments (Fig. 7). This data confirmed that CerP could potentially be a marker for discrimination of urinary exosomes from urinary microvesicles.

**Figure 7:** Validation of the lipidomics data using dot blot analysis. Dot blot analysis was performed to validate the presence of CerP only in urinary exosomes, but not in urinary microvesicles. The full-length images of these cropped dot blots are provided in Supplementary Fig. S2. MV = microvesicles; Exo = exosomes.

## Discussion

For biogenesis, exosomes are specifically originated from an invagination of endosomes that subsequently fuse with multivesicular body (MVB) and finally expel from the cells^5,9^. During the invagination process, which is mainly regulated by endosomal sorting complex required for transport (ESCRT) protein complexes, cytosolic proteins, mRNAs and micro RNAs (miRNAs) are engulfed into the intraluminal vesicle^10^. Exosomes are released from the cell to the extracellular space by fusion of MVB with the inner membrane of the parental cell^9,11^. By contrast, microvesicles are originated by direct budding of the plasma membrane from the parental cell^12^. The budding mechanism of microvesicles are regulated mainly by intracellular calcium level^13^. High concentration of calcium ion leads to calpain activation, exposure of phosphatidylserine at the outer membrane, disruption of cytoskeletal assembly, and outward protrusion of plasma membrane to form the microvesicles^14^.

Recently, protein and lipid compositions of exosomes and microvesicles have been broadly and extensively investigated to better understand their biology and to define biomarkers for their clear distinction^15–20^. Regarding lipid contents, a previous study has reported that the enrichment of particular lipid types of exosomes and microvesicles is related to their biogenesis^21^. Comparing to their parental cells, exosomes have been proposed to be enriched with sphingolipids involving MVB formation, whereas microvesicles are enriched with phospholipids, including phosphatidylethanolamine and phosphatidylserine corresponding to the lipid compositions of plasma membrane^15–20^.

Lipids play several pivotal roles in fundamental biological functions of EVs, including cell membrane structure, chemical signaling and cholesterol metabolism^20^. Generally, membrane-bounded vesicles derived from mammalian cells are composed of five major classes of lipids, including sphingolipid, fatty acid, glycerolipid, glycerophospholipid and sterol lipid classes^22^. Each of these lipid classes contain the diversity of lipid species^22^. Lipid species can be defined by transformation of head and tail groups, which may contain various modifications^23^. With such modifications, complexity and heterogeneity of these lipids are increased in each biological membrane^24^. Nevertheless, the precise information of distinct lipid compositions of microvesicles and exosomes remained unclear and needed elucidations.

In the present study, MALDI-TOF MS revealed that the lipidome profile of urinary microvesicles obviously differed from that of urinary exosomes. Additionally, urinary exosomes seemed to have more lipid species, in particular sphingolipids, as compared to urinary microvesicles. It may be possible that urinary exosomes contain greater proportion of lipid species with higher heterogeneity and complexity than those of microvesicles^25^. Furthermore, the data also implicate that such lipid species are essential for exosomal formation during biogenesis via ceramide-dependent pathway^25^.

Interestingly, CerP was detectable only in urinary exosomes. We could validate such obvious difference in urinary exosomes vs. microvesicles using dot blot analysis. Moreover, overall ceramides (Cer) had greater levels in urinary exosomes. Ceramide lipid species is synthesized by hydrolysis of the phosphocholine moiety of sphingomyelin by the function of shingomyelinase^26^ and acts as the second messenger during response to various stimuli or stresses^27^. Ceramide has been proposed to get involved in MVB formation and in sorting of the ubiquitinated proteins to exosomes^28^. Specifically, ceramide is the cone-shaped structure lipid that facilitates invagination of intraluminal vesicle in MVB^25^. In previous studies, treating the cells with a sphingomyelinase inhibitor resulted in the reduction of ceramide production and subsequently the decrease of exosomal secretion from the cells^18,29^. In addition to ceramides, our present study also showed the enrichment of HexSph and LacCer, other species in the sphingolipid class, in urinary exosomes as compared to urinary microvesicles. These data were consistent with the results obtained from a previous study indicating that these sphingolipids were also enriched in exosomes when compared to their parental cells originated from prostate cancer^17^.

Although the data obtained from this study were interesting and could be confirmed by another conventional method, technical limitations should be noted. Our MALDI-TOF MS data showed that several lipid species were identified from the same TLC band and, on the other hand, some of the same lipid species were identified from different TLC bands. Due to the complexity in physicochemical properties of lipids (e.g., acyl long chain, head group and unsaturated bonds), our TLC protocol might not be able to completely resolve each of the lipid classes in the mixture that tended to co-migrate along the limited length of the TLC plate^30,31^. As also demonstrated in our present study, several species of sphingolipid, fatty acid, glycerolipid and phospholipid classes seemed to be co-eluted in both mobile phases using 65:24:4 (by volume) chloroform/methanol/water and 5:2:4:2:1 (by volume) chloroform/methanol/acetone/acetic acid/water. Therefore, using the higher-resolution TLC protocols may reduce such redundancy. In addition, only MALDI-TOF MS (which is a fingerprinting technique) was employed for the identification of lipid class/species in the present study. Using a higher-resolution MS model, e.g., LIFT (laser ionization fragmentation technology) TOF/TOF tandem MS (MS/MS), would yield more accurate results.

In addition to the technical issues mentioned above, other factors might also contribute to the redundant lipid identification on different TLC bands. A previous study has reported that ceramide containing non-hydroxy fatty acids and sphingosines (CerNS) with different numbers of carbon atoms at acyl side chain could be found in two TLC spots^32^. Similarly, another study has also shown that CerNS containing greater number of carbon atoms at the acyl side chain was resolved as the upper TLC band, whereas CerNS with smaller number of carbon atoms at the acyl side chain was present as the lower bands^33^. These data suggest that difference in the length of the acyl side chain has an impact on chromatographic migration of the lipid species^32,33^. Furthermore, type of the functional group conjugated with the acyl side chain of the lipid species can affect the TLC lipid separation. For example, triacylglycerol (TAG) containing one, two or three hydroxyl groups could be resolved as the different TLC bands^34,35^. Finally, modification within the side chain can also affect the TLC separation of the lipid species as in the case of PC with various oxidation characteristics that were resolved as different TLC bands^36^. In our present study, only MALDI-TOF MS was employed to identify the lipid class/species. Because this fingerprint technique is unable to precisely discriminate the same lipid species with varieties in side-chain lengths, conjugated functional groups and modifications, the higher-resolution MS, such as LIFT-TOF/TOF MS, is required for such precise discrimination.

In summary, we report herein the distinct sphingolipid profiles of urinary microvesicles vs. exosomes. CerP, HexSph, LacCer, M(IP)2 C, SHexCer and SHexSph were detectable only in urinary exosomes, whereas PI-Cer were detectable only in microvesicles. The presence of CerP only in urinary exosomes was successfully validated by dot blot analysis. Our extensive lipidome analyses of urinary microvesicles vs. exosomes provide potential lipidome markers to discriminate exosomes from microvesicles and may lead to better understanding of EVs biogenesis.

## Materials and Methods

### Urine collection and processing

This study was approved by the institutional ethical committee (Siriraj Institutional Review Board) (approval no. Si650/2015). All the experiments involved human subjects and clinical samples were conducted according to the international guidelines, i.e. the Declaration of Helsinki, the Belmont Report, and ICH Good Clinical Practice, and informed consent was obtained from all subjects. The urine collection was performed according to previous studies^37,38^. Briefly, mid-stream urine samples were collected from 8 healthy individuals (2 males and 6 females). An equal volume from each urine sample was pooled and then centrifuged at 1,000 *g* and 25 °C for 10 min to remove cellular debris and particles. Clear supernatant was collected and further processed for isolation/purification of microvesicles and exosomes.

### Isolation/purification of urinary microvesicles and exosomes

Urinary microvesicles and exosomes were isolated by differential centrifugation as described previously^39,40^. Briefly, the clear supernatant of each urine sample was centrifuged at 10,000 *g* and 4 °C for 30 min to isolate urinary microvesicles. Thereafter, urinary exosomes remained in the supernatant were isolated by an ultracentrifugation at 100,000 *g* and 4 °C for 90 min using an ultracentrifuge (Sorvall; Langenselbold, Germany). After isolation, microvesicles and exosomes were resuspended in 200 µl PBS for lipid extraction.

### Transmission electron microscopy (TEM)

Examination of urinary EVs using TEM was performed according to protocols reported previously with slight modifications^39,40^. Briefly, the isolated/purified microvesicles or exosomes were resuspended in 2% (w/v) paraformaldehyde and loaded onto carbon-Formvar-coated copper grids (EMS; Hatfield, PA). The samples were left on the grids for 20 min to adsorb and form monolayers. The grids were then washed three times with 100 µl PBS, fixed with 50 µl of 2% (v/v) glutaraldehyde for 5 min and subsequently washed eight times with distilled water. The grids were contrasted with 50 µl of 4% (v/v) uranyl acetate (pH 7.0) for 10 min and the excess fluid was removed by filter paper. The grids were left to air-dry for 10 min and then loaded onto a transmission electron microscope (Tecnai G2 TEM Series; Hillsboro, OR) with an accelerating voltage set at 80 kV and original magnification of 50,000 × . All images were captured using slow-scan CCD camera (FEI Eagle CCD Camera; Hillsboro, OR).

### Lipid extraction

Lipids from urinary microvesicles and exosomes were extracted using protocol described previously with slightly modification^41^. Briefly, 600 µl of 2:1(v/v) chloroform/methanol (Fisher Scientific; Loughborough, UK) was added into 200 µl of suspension containing microvesicles or exosomes (isolated/purified from 300 ml pooled urine) and mixed at 25 °C for 15 min. Separation of organic solution into two phases was performed by adding 100 µl deionized water, mixed for 1 min and centrifuged at 1000 *g* and 20 °C for 15 min. The organic phase containing lipids (lower layer) was collected using a pipette and transferred into a new tube. The lipid extract was then dried in a SpeedVac concentrator (Savant; Holbrook, NY). The dried lipids were weighed to determine the lipid amount derived from microvesicles or exosomes.

### TLC separation

The extracted lipids with an equal amount of 10 µg/sample were resuspended in 10 µl of 2:1(v/v) chloroform/methanol and then resolved by TLC. For an initial stationary phase, the sample was applied onto the starting line of TLC silica matrix plate (Sigma-Aldrich; St. Loius, MO). Thereafter, the sample separation was run in the first mobile phase using 65:24:4 (by volume) chloroform/methanol/water with 6-cm distance in the saturated glass chamber at 25 °C for 15 min. The sample was then subjected to the second mobile phase using 5:2:4:2:1 (by volume) chloroform/methanol/acetone/acetic acid/water at 25 °C for 15 min. Finally, the TLC plate was dried at 25 °C for 5 min. Visualization of the resolved lipid bands was done using iodine vapor in a closed chamber for 30 min and their images were captured by a ChemiDoc MP Imaging System (Bio-Rad; Berkeley, CA).

### Lipidome profiling and identification by MALDI-TOF MS

Each of the TLC bands visualized from microvesicular or exosomal sample was scrapped from the silica plate, resuspended in 2:1(v/v) chloroform/methanol and analyzed using UltrafleXtreme MALDI-TOF/TOF mass spectrometer (Bruker Daltonik; Bremen, Germany) as previously described^41^. Briefly, the TOF was calibrated using a peptide mixture (Bruker Daltonik) before acquisition of the sample spectra. Equal volume (1–2 µl) of lipid extract and MALDI matrix solution (0.5 M 2,5-dihydroxybenzoic acid in methanol containing 0.1% trifluoroacetic acid) was mixed in a 0.6-ml microcentrifuge tube. Then, 1 µl of the mixture was spotted onto a MALDI plate. The mass spectra were acquired over the *m/z* range of 0–2,000 in positive ion Reflectron TOF mode. The laser power was adjusted to a point just above the ionization threshold of the sample, and the laser rate was set at 10 Hz with 1,000 laser shots per acquisition. A total of 10 acquisitions were averaged for each sample.

### Data analysis

The mass lists and intensities were obtained by peak detection algorithm within FlexAnalysis software (Bruker Daltonik). Signal to noise threshold of 4, peak width of 0.1 *m/z*, and Tophat base line subtraction were used as the default parameters. The *m/z* values of lipid ions were searched against LIPID MAPS Structure Database (LMSD) using the LIPID MAPS tool (www.lipidmaps.org/tools). The [M + H]^+^ and [M + Na]^+^ were selected in the positive ionization mod. The mass tolerance was set at ± 0.2 Da. Lipid categories were limited to major lipid classes commonly found in membrane organelles, including fatty acids, glycerolipids, glycerophospholipids, sphingolipids and sterol lipids. The relative intensity of each lipid species identified was normalized by total intensity of all lipid species found in each sample.

### Validation by dot blot analysis

Lipids derived from urinary microvesicles or exosomes with an equal amount (5 µg in 5 µl of 2:1(v/v) chloroform/methanol) were dotted onto a nitrocellulose membrane (Whatman; Dassel, Germany) and then allowed to air-dry. Non-specific bindings were blocked with 5% (w/v) skim milk in PBS at 25 °C for 1 h. After washing, the membrane was incubated with biotinylated anti-human ceramide-1-phosphate antibody (MyBioSource; San Diego, CA) at a dilution of 1:1,000 in 1% skim milk/PBS at 4 °C overnight. After washing with PBS three times, the membrane was then incubated with streptavidin conjugated with horseradish peroxidase (MyBioSource) (1:2,000 in 1% skim milk/PBS) at 25 °C for 1 h. Immunoreactive dot was then developed with SuperSignal West Pico chemiluminescence substrate (Pierce Biotechnology; Rockford, IL) and then visualized by autoradiogram.

## Supplementary information

Supplementary Figures S1-S2 and Tables S1-S2
